# Status of Bioinformatics Education in South Asia: Past and Present

**DOI:** 10.1155/2021/5568262

**Published:** 2021-04-26

**Authors:** Muhammad Muddassir Ali, Muhammad Hamid, Muhammad Saleem, Saadia Malik, Natash Ali Mian, Muhammad Ahmed Ihsan, Nadia Tabassum, Khalid Mehmood, Furqan Awan

**Affiliations:** ^1^Institute of Biochemistry and Biotechnology, University of Veterinary and Animal Sciences, Lahore 54000, Pakistan; ^2^Department of Statistics and Computer Science, University of Veterinary and Animal Sciences, Lahore 54000, Pakistan; ^3^Department of Industrial Engineering, Faculty of Engineering-Rabigh, King Abdulaziz University, Jeddah 21589, Saudi Arabia; ^4^Department of Information Systems, Faculty of Computing and Information Technology-Rabigh, King Abdulaziz University, Jeddah 21589, Saudi Arabia; ^5^School of Computer and IT, Beaconhouse National University, Lahore 54000, Pakistan; ^6^Faculty of CS and IT, Virtual University of Pakistan, Lahore 54000, Pakistan; ^7^Faculty of Veterinary and Animal Sciences, The Islamia University of Bahawalpur, 63100, Pakistan; ^8^College of Veterinary Medicine, South China Agricultural University, Guangzhou 510642, China

## Abstract

Bioinformatics education has been a hot topic in South Asia, and the interest in this education peaks with the start of the 21^st^ century. The governments of South Asian countries had a systematic effort for bioinformatics. They developed the infrastructures to provide maximum facility to the scientific community to gain maximum output in this field. This article renders bioinformatics, measures, and its importance of implementation in South Asia with proper ways of improving bioinformatics education flaws. It also addresses the problems faced in South Asia and proposes some recommendations regarding bioinformatics education. The information regarding bioinformatics education and institutes was collected from different existing research papers, databases, and surveys. The information was then confirmed by visiting each institution's website, while problems and solutions displayed in the article are mostly in line with South Asian bioinformatics conferences and institutions' objectives. Among South Asian countries, India and Pakistan have developed infrastructure and education regarding bioinformatics rapidly as compared to other countries, whereas Bangladesh, Sri Lanka, and Nepal are still in a progressing phase in this field. To advance in a different sector, the bioinformatics industry has to be revolutionized, and it will contribute to strengthening the pharmaceutical, agricultural, and molecular sectors in South Asia. To advance in bioinformatics, universities' infrastructure needs to be on a par with the current international standards, which will produce well-trained professionals with skills in multiple fields like biotechnology, mathematics, statistics, and computer science. The bioinformatics industry has revolutionized and strengthened the pharmaceutical, agricultural, and molecular sectors in South Asia, and it will serve as the standard of education increases in the South Asian countries. A framework for developing a centralized database is suggested after the literature review to collect and store the information on the current status of South Asian bioinformatics education. This will be named as the South Asian Bioinformatics Education Database (SABE). This will provide comprehensive information regarding the bioinformatics in South Asian countries by the country name, the experts of this field, and the university name to explore the top-ranked outputs relevant to queries.

## 1. Introduction

Bioinformatics is an emerging discipline, and with its advancements, there will be more opportunities for scientists in applied and pure research [1–5]. Nowadays, bioinformatics or computational biology has extreme prospect in genomic analysis and complete protein studies. Bioinformatics created a new community by maintaining networks among different areas and allow the researcher to work peacefully with the support of the whole community on its back. The cost of running the bioinformatics laboratory equipment and its teaching is far less than running molecular techniques and equipment. In bioinformatics, we mostly deal with software, algorithms, tools, and databases to perform the analysis of a desired sample.

European countries, USA, and UK are taking the lead in the field of bioinformatics [6–10]. South Asian countries are developing countries with immense pace; however, these bioinformatics fields are not much developed. Bioinformatics is a complex multidisciplinary field that analyzes and develops tools to manage and store the continuous growing biological data. This led to increase the importance and the efficiency of bioinformatics education in performing research [7, 11–14].

So, it is pertinent to take an overview of bioinformatics education in South Asia keeping in mind the diverse geographical and geopolitical situation of these countries. The current review would provide the current status of bioinformatics education, challenges, and development for the bioinformatics in South Asian countries. This would help to formulate policies for future development in the field of bioinformatics with more precision and insight.

The rest of the paper is organized as follows: in Section 2, history of bioinformatics in South Asia is discussed. The universities offering bioinformatics are described in Section 3. In Section 4, the bioinformatics curriculum in South Asia is presented. In Section 5, the bioinformatics conferences and workshop in South Asia are described in detail while Section 6 highlights the opportunities for bioinformatics in South Asia. In Section 7, the challenges the bioinformatics is facing in South Asia are defined while Section 8 describes the comprehensive platform framework for the development of South Asian Bioinformatics Education Database. In Section 9, suggestions for the improvement of bioinformatics education in South Asia is presented while Section 10 concludes the research and provides directions for future work.

## 2. History of Bioinformatics in South Asia

India is the first country among all the South Asian countries to introduce a formal study in bioinformatics. With the establishment of a nationwide network of distributed information centers (DICs) under the support of the Indian government and biotechnology information system (BTIS), India started the formal bioinformatics activities in the early 1980s [15, 16]. During the early years, generalized and short-term training programs were conducted in different areas of bioinformatics. In the 1980s, the main purpose of training programs was to build awareness of bioinformatics among IT professionals, biologists, and mathematicians [14, 16–18]. In the coming years, these training programs will be evolved and will give more theme-based training on topics like biological database, database searches, algorithms and their applications, and structural bioinformatics and simulations. From the beginning of the new millennium, these DICs expanded their bioinformatics domain and started working on different bioinformatics aspects like genomics, proteomics, structural bioinformatics, and other domains [19–21].

COMSATS Institute of Information Technology (CIIT) and Muhammad Ali Jinnah University are the pioneers to introduce a bioinformatics study in Pakistan in 2003 [22]. Later, many other universities introduced bachelor's degree programs in this discipline, such as International Islamic University, Government College University, and University of Veterinary and Animal Sciences. From 2003, many workshops and conferences were conducted by the Higher Education Commission (HEC) of Pakistan on bioinformatics in institutions like Centre for Excellence in Molecular Biology (CEMB) and CIIT. In 2010, Regional Science Group Pakistan (RSG-P) was established, with a motto to change the scientific environment in Pakistan via knowledge sharing in computational science and in bioinformatics. RSG-P provided a platform for a bioinformatician to share their thoughts to enhance the prospect of bioinformatics in Pakistan [22].

Bangladesh is a young and prospective country on biological research especially on bioinformatics. As for now, there is not a single university in Bangladesh that has well-developed multidisciplinary bioinformatics course that incorporates most public-domain databases, research tools, peer-review journals, and research organizations. However, there are universities present in Bangladesh which offer bioinformatics study which helped a lot in pharmaceutical and biotechnological industry. The continuous progress of information and communication technology (ICT) had already laid the basis of bioinformatics studies and biological data analysis in Bangladesh. Bangladesh's pharmaceutical industry now meets 96 percent of the country's pharmaceutical needs [23], mainly because of extensive governmental funding in the pharmaceutical industry. The government of Bangladesh started offering a course combining pharmaceuticals with bioinformatics to promote and create awareness of bioinformatics within the country [23]. This helps to develop and stabilize companies for bioinformatics and pharmaceutical side by side.

In Nepal, two institutes teach bioinformatics to students. In 2003, the Department of Biotechnology at Kathmandu University started introductory courses on bioinformatics [24]. In 2012, Nepal acquired its first research database [25]. The database lacks expressed sequence tag (EST) records and genome survey sequenced record (GSS).

In Sri Lanka, bioinformatics came in between 2002, when the Department of Plant Sciences at the University of Colombo introduced a special course by the name of “Introduction of Bioinformatics.” In 2010, four Sri Lankan universities started teaching bioinformatics. Currently, there is no government-made database of bioinformatics; however, the government organized many conferences and diplomas to increase the awareness of bioinformatics [26].

## 3. Universities Offering Bioinformatics

In India, more than a hundred universities are offering bioinformatics degree at different graduation and postgraduation levels [16, 26–28]. Details of some universities are provided in Table 1 (see Supplementary File) which includes a complete description about the universities' web link and the programs being offered.

In Pakistan, around thirty universities are offering bioinformatics as a professional degree [29]. A list of some universities along with their details of the courses is presented in Table 2 (see Supplementary File).

The study of bioinformatics is quite expensive in Sri Lanka. There are few institutes in Sri Lanka where bioinformatics is taught at the undergraduate level while only one university started offering bioinformatics at the Ph.D. doctorate level. Sri Lanka has currently more than 16 persons holding a Ph.D. degree in bioinformatics. Table 3 (see Supplementary File) furnishes details of the university which is presently offering bioinformatics degrees and courses in Sri Lanka [26].

In Nepal, bioinformatics was introduced in 2003. Nepal has only two institutes that are offering study in bioinformatics. A major factor for the late start of bioinformatics in Nepal is her landlocked geographical location on the world's map, and besides that, Ph.D. professors of bioinformatics are not in a collaboration with each other.

In Bangladesh, currently, three institutions are offering degree in bioinformatics, but progress is being made by the government of Bangladesh to make more institutes for biological sciences especially biotechnology and bioinformatics [25]. Table 4 (see Supplementary File) presents details of universities, which are offering bioinformatics in Nepal and Bangladesh.

The other countries of South Asia like Afghanistan, Bhutan, and Maldives are currently having no institution regarding the study of bioinformatics.

## 4. Bioinformatics Curriculum in South Asia

### 4.1. Diploma

The first diploma in bioinformatics was started in India during the year 2000. At first, biotechnology information system started an advanced diploma in bioinformatics in Jawaharlal Nehru University, University of Pune, University of Calcutta, Pondicherry University, and Madurai Kamaraj University [30]. Like India, Pakistan also started a one-year diploma in 2002 at the Pakistan Institute of Modern Sciences and Virtual University (VU) of Pakistan. In Nepal, the Department of Biotechnology started a one-year diploma in 2003 at the University of Kathmandu [24, 31].

The scheme of studies for a diploma is quite smooth and specially designed for those students who completed their bachelor in either basic science or medicine. The aim of these diploma programs is to build the awareness of bioinformatics among the student of natural science and to level the field for the introduction of undergraduate and postgraduate studies in South Asia especially.

### 4.2. Bachelors

Based on educational and industrial needs, every South Asian country varies in the curriculum of bioinformatics. In India, a bachelor's degree has various names, like B.Tech, BSc, M.Sc., and BS. The BSc and M.Sc. combine have worth equal to the four-year bachelor, while BS and B.Tech itself have a four-year program [32].

In Pakistan, Bangladesh, Nepal, and Sri Lanka, there is no concept of BSc; all universities offer only BS Hons program. Institute of Bioinformatics in India, COMSATS CIIT in Pakistan, the University of Kathmandu in Nepal, and the University of Colombo in Sri Lanka are some of the best institutes for bioinformatics study [29, 32, 33].

### 4.3. Masters

The University of Pune was the first university to start a master's degree program in bioinformatics in South Asia, with the financial support of the Department of Biotechnology (DBT) in 2002. During the early years, research or thesis was optional for masters in bioinformatics but now, it has become compulsory. In India alone, more than 29 universities are offering a master's degree in bioinformatics and the present curriculum has evolved from only theoretical bases to the research-oriented one. In Pakistan, 9 universities are offering masters in bioinformatics. Nepal, Sri-Lanka, and Bangladesh have only 1 university offering a master's degree in bioinformatics. Most South Asian universities are offering 90 credit hours for master's degree in bioinformatics. Research and thesis are now compulsory to get a degree in most South Asian institutes [19]. The master's level courses of bioinformatics in South Asia are specially designed to meet the local industry demands. The master's degree is more focused on the specific domain of bioinformatics like algorithms for the database and molecular biology, protein structure analysis, and microarray data.

### 4.4. Ph.D.

In 1997, the University of Pune was the first institute throughout South Asia to start a Ph.D. in bioinformatics. The University of Pune is also the first university in South Asia to award a Ph.D. in bioinformatics in 2003. Currently, there are many public and private universities in India which are offering Ph.D. in bioinformatics like Indian Institute of Technology (IIT), National Centre for Biological Science (NCBS), Center for Cellular and Molecular Biology (CCMB), and National Institute of Pharmaceutical Education and Research (NIPER). These Ph.D. programs are funded by multiple institutes like DBT, Department of Science and Technology (DST), Ministry of Communication and Informational Technology (MCIT), and University Grant Commission (UGC) [34, 35].

In Pakistan, only 3 universities are offering a doctoral-level study in bioinformatics. Quaid-e-Azam University (QAU) was the first university in Pakistan which started offering a Ph.D. in bioinformatics while the other two universities are Hazara University and Capital University of Science and Technology. Ph.D. in bioinformatics was started in 2008 in Pakistan. There are many organizations that grant funding and support to bioinformatics' students. HEC of Pakistan is the biggest supporting organization; others include National Center for Bioinformatics (NCBI), Bioinformatics Research Lab (BRL), and Institute of Molecular Science and Bioinformatics (ISMB) [31, 36].

Asian University for Women is the only university in Bangladesh which started offering a Ph.D. in bioinformatics in 2009. Bangladesh Bioinformatics and Computational Biology Association (BBCBA), Molecular Modelling and Drug Design Laboratory (MMDDL), and Bangladesh Council of Scientific and Industrial Research Laboratories (BCSIR) are the few institutes that deal with bioinformatics in Bangladesh.

Department of Biotechnology of Kathmandu University is the only department in Nepal which is offering Ph.D. in bioinformatics with the collaboration of some foreign organizations.

In Sri Lanka, Ph.D. in bioinformatics was started in 2013. The University of Colombo and the University of Peradeniya are two universities which are offering a Ph.D. degree in bioinformatics.

## 5. Bioinformatics Conferences and Workshop in South Asia

There are many steps taken by the HEC, and many teaching activities are in process since 2003. From 2003, the HEC supported financially on organizing conferences, committees, and conferences on bioinformatics. These workshops and conferences are organized by highly ranked institutes such as CIIT/COMSAT Islamabad, CEMB, and Punjab University Lahore. The major importance of these conferences and workshops is the interaction of local researchers with foreign or other local researchers and the transfer of new innovative ideas. Table 5 (see Supplementary File) provides information about workshops, symposiums, and conferences that were held in South Asia. Almost more than 33 workshops and conferences have been organized by the government of Pakistan and many universities to promote the awareness of bioinformatics and its applications among people in society. India is leading the race of bioinformatics in South Asia. Many conferences and workshops have been organized to enhance the promotion and knowledge of bioinformatics among Indians. Almost more than 100 conferences and workshops in the last 5 years had been organized in India just to increase the interaction of local researchers with the international researcher to discuss new topics and transfer of knowledge. The major aim of the Indian government is to comply with or attract foreign investors in India for the improvement of the native bioinformatics industry and market. Sri Lanka, Bangladesh, and Nepal had few conferences and workshops in the past years, but their motives and ideas had been reforming; therefore, almost 3 conferences on bioinformatics were organized by Bangladesh in this year [37]. The way of bioinformatics is soothing in these developing countries, and thus, it helps to advance their native technology regarding natural sciences. Few conferences and their descriptions are given below; the rest of the details: titles, organizers, and dates about conferences and workshops, are furnished in Table 5 (see Supplementary File).

### 5.1. Pre-18th FAOBMB Symposium Satellite Workshop on Bioinformatics, Pakistan

This symposium was held in the CEMB, Lahore, Pakistan, between 14^th^ November and 19^th^ November 2005. This conference is sponsored by different organizations like CEMB, Federation of Asian and Oceanian Biochemists and Molecular Biologists, APBioNet, and Progeniq Pte Ltd. This symposium is organized with the aim of bringing Pakistan's bioinformatics community together, understanding new bioinformatics concepts, and providing platforms for researchers, professors, and students to discuss certain issues. Five professors and scientists from Sweden and Singapore participated in this symposium.

### 5.2. Advances in Bioinformatics in the Postgenomic Era Workshop, Pakistan

The workshop was conducted in the National Center for Bioinformatics (NCBI) of QAU [34]. This workshop was sponsored by QAU, and the major aim of this workshop was to introduce new technology and strategies about bioinformatics in genomics and proteomics to train young scholars for the techniques which emerge in the bioinformatics field. All scholars and lecturers were from Pakistani universities.

### 5.3. Bioinformatics Workshop Hands-On Training on Analysis of Biological Data Using R, Pakistan

This workshop was held at VU on 5^th^ January 2016. The workshop was sponsored by the VU and HEC [38]. The workshop had an aim to relate two different fields like bioinformatics and statistics to produce more perfect results, introducing R techniques which can be utilized in bioinformatics and building fundamental skills. All scholars, professors, and scientists in this workshop were from Pakistani universities like VU, COMSAT, CEMB, and QAU.

### 5.4. Computational Biology Workshop, Pakistan

This workshop was conducted by Habib University from 31st July to 4th August 2017. This workshop was sponsored by many private companies along with the university itself. The aim of the workshop was to provide information about computational techniques, how these techniques will communicate with biology, and the principle of biology and current affairs of research conducted in this field. Scholars and professor participated in this workshop were from America, Australia, UK, and Pakistan [38].

### 5.5. Indian Conference on Bioinformatics 2017 (Inbix')

This conference was organized by http://Bioclues.org/ in association with Birla Institute of Scientific Research (BISR) in Jaipur, Rajasthan, India. BISR hosted this conference from 07 to 09 November 2017. This international conference was organized with the hope to foster the interactions and collaborations among young researchers and to connect them with the top researchers in the bioinformatics and computational biology. Temple-Smith from Boston University and Thomas Sicheritz from Technical University of Denmark were the keynote speakers at this conference [34].

### 5.6. Bifx India Virtual Conference 2010

Bifx India Virtual Conference was the first of its kind in India. It was organized by http://Bioclues.org/ with the support of Bioinformatics Organization of India, Asia Pacific Bioinformatics Network (APBioNet), and International Society for Computational Biology. The date of this conference was the 12^th^ and 13^th^ of February 2010. Dr. Søren Brunak (Denmark Technical University), Dr. Thomas Knudsen (National Center for Computational Toxicology, EPA, United States), Dr. Shoba Ranganathan, (Macquarie University, Australia), Dr. David Reif (National Center for Computational Toxicology, EPA, United States), Dr. Russel Thomas, (The Hamner Institute, United States), and Dr. Tin Wee Tan (National University of Singapore, Singapore) were the keynote speakers of this conference.

### 5.7. The Eighth Asia Pacific Bioinformatics Conference, India

The 8^th^ Asia Pacific Bioinformatics Conference was held in the Indian Institute of Science, Bangalore, from January 18 to 21, 2010. The conference focused on the following topics which are sequence analysis, motif search/analysis, RNA analysis, physical and genetic maps, evolution and phylogeny, protein structure analysis, transcription, gene expression, proteomics, and population genetics/SNP/haplotyping.

### 5.8. International Conference on Bioinformatics (ICBINF-18), Sri Lanka

Research League of Sri Lanka has organized an international conference on bioinformatics in Kandy, on the 12th of October 2018. The aim of this conference was to provide a platform to the researchers and practitioners from both academia and industry to share cutting-edge development in the field of bioinformatics.

## 6. Opportunities for Bioinformatics in South Asia

Bioinformatics gained importance due to its advancements; there will be more opportunities for scientists in applied and pure research. The cost of running the bioinformatics laboratory equipment and its teaching is far less than running molecular techniques and equipment. Most of the bioinformatics software is freely available on the internet for academic purposes. The main perspective of bioinformatics is to store lots of biological data in the form of a database. The development of new standards and software coding rules would ease our way to conduct research by helping us to analyze and match the preexisting genomic data. The availability of good services for data deposition, good programming, and data analysis would gain much importance in bioinformatics to remove false data from databases.

India has a well-developed system of biotechnology as compared to other South Asian countries based on business to business (B2B) structure where it provides services to business. With the help of biotechnology, pharmaceutical and agriculture industries are changing the lives of local communities. The government of India has taken serious efforts to introduce bioinformatics in its universities which really helps India to increase its revenue in the global bioinformatics market. The advances in the field of bioinformatics and the pharmaceutical industry would be a huge bonus for India. The government of India has systematic effort in bioinformatics industry and research if it can properly capitalize on its resources. IT companies like Infosys, Cognizant Technology, and Tata consultancy services (TCS) are now investing in computational biology along with other IT services. The Indian government and bioinformatics companies can look forward to bioinformatics services like deoxyribonucleic acid (DNA) mapping, DNA mining, DNA sequencing, and functional gene analysis. Biotechnology information system (BTIS) along with DBT is promoting bioinformatics and recently developed a Bio-IT Park. Bioinformatics in India has gained significant growth by information technology and institutional education. Biotechnology information system network (Bitnet) has developed a countrywide network that provides valuable information to students and experts in biotechnology and bioinformatics. These databases offer the students an opportunity to learn about processing, efficient organization, formatting of data, gene mapping, gene identification, new genes, and protein analysis. These networks and industries provide enormous job vacancy for bioinformaticians and also provide new innovative ideas to students to perform an industry-oriented and profitable research. Being the largest English-speaking scientific workforce in the world, we are hopeful that a lot of opportunities would come to India and Pakistan in the coming years [36].

Although the development capability and jobs of bioinformatics in Pakistan are less than in those India, still, it has a large potential for bioinformatics to prosper. Most of the Pakistani students graduated in bioinformatics are working either in academia or in pharmaceutical industries. Many types of bioinformatics jobs are available in Pakistan for the computational specialist as either implementation of system and program for management or analysis and storage of a vast amount of sequence DNA. The laboratory information management systems (LIMS) major objective is to improve the accuracy of results, to ease the access to databases, and to increase the utilization of data. RSG-P provides a forum for local bioinformaticians to collaborate with other students, experts, and academicians. It would provide an opportunity to uplift research in bioinformatics. Every lab requires qualified bioinformaticians to perform dry work and run their confirmatory tests. Development of EMBnet and e-book helped to develop a database for local students to add their research for the promotion of bioinformatics in Pakistan. There is an increasing opportunity for bioinformatics students in the pharmaceutical industry in drug development and disease control. As Pakistan is an agricultural country and most of the research work is done on plants and agriculture by agriculturists and plant biotechnologists, bioinformatics assists in this particular area to increase the workflow and this will promote the bioinformatics and cause vacancy of jobs in this particular area.

Due to its unique fauna and flora, Nepal is one of the most prospective places for biologists. There is a huge possibility that bioinformatics can get interesting information from the species of Nepal as most of them are biologically undiscovered. Every country needs computational data to conserve its natural resources, and bioinformaticians are the only data analysts present to analyze data with biological knowledge. In short, we can say that bioinformatics has a huge scope in agriculture and medical health in Nepal.

Bangladesh is still new in bioinformatics research. Bangladesh has no infrastructure for bioinformatics, and no university is well developed. However, recently, a Bangladeshi research group had developed a global network and introduced important research areas to talented researchers and students. Bangladeshi bioinformaticians would allow the pharmaceutical companies to gain new achievements and increase efficiency rate by the introduction of new tools and designs and new screening test; this provides more jobs and more learning for students. A large number of vacancies are empty for bioinformaticians in the pharmaceutical industry to organize and analyze biological data. However, unfortunately, there is no one to fill them.

In Sri Lanka, the opportunity for bioinformaticians is increasing day by day as the government has started an awareness program by combining forces with the University of Colombo and added one seat of bioinformatician in every hospital and research lab which collects and analyze the biological data. Sri Lanka also has a journal to publish local bioinformatics work with the name of *Sri-Lanka Journal of Bio-Medical Informatics* [36].

## 7. Challenges That Bioinformatics is Facing in South Asia

Being an integrated science, bioinformatics faces many challenges and problems in South Asia. Biology experts have no expertise in computer functioning, programming, and computer theories. Another major problem in South Asia is the lack of experts in bioinformatics. Governments sent people to foreign countries to acquire knowledge for the country, but most of them never returned [29, 33]. Some of the challenges that South Asian countries are facing to improve the status of bioinformatics are as follows.

### 7.1. Education Quality

The bioinformatician must have an understanding of biology, statistics, computer science, IT, and mathematics along with core bioinformatics knowledge. Only a handful of teachers with expertise enlisted above are available for teaching and research in South Asia. Although new universities are opening every year, still, academia is unable to produce well-trained bioinformaticians in South Asia [27, 29]. In India, an average of 35 persons are getting their Ph.D. degrees in bioinformatics every year, while in Pakistan, an average of 12 persons get their Ph.D. degree in bioinformatics. In Sri Lanka, there are only 16 Ph.D. scholars so far and most of them migrated to foreign countries. This brain drain is the main reason behind the shortage of teachers and experts in bioinformatics.

### 7.2. The Gap between Biological and Computer Sciences

Biology and computer sciences are two different fields, and both have different perspectives and scope. The biologist generally does not know about the deep understanding of computer science, and computer experts lack knowledge in biology. Understanding the concepts of both fields of study is a tiresome process, and sometimes, biologists face failure just because they are not able to communicate their ideas to IT experts or vice versa. There is not even a single algorithm made by experts from Pakistan, India, Nepal, or Bangladesh. In 2014, HEC, BTIS, and BBCBA planned a scheme to add bioinformatics as a compulsory subject in all biology and natural science degrees aimed at improving the student extinct toward bioinformatics.

### 7.3. Learning Method and Education

In India, more than 90 institutes are teaching bioinformatics at bachelor's, master's, or Ph.D. levels, but unfortunately, a number of application-oriented students are far less than the desired amount. In Pakistan, the major problem is the curriculum. From 2003 to 2014, HEC amended the curriculum of bioinformatics eight times. On the basis of the multidisciplinary nature of the subject, multiple methods were applied to achieve the desired outcome. Courses regarding the programming skills were also enhanced. Adaption to teach bioinformatics is also a problem because teaching bioinformatics is enormously different from teaching other natural science degrees [29, 30, 33].

### 7.4. Lack of Algorithm Development

India is considered an IT hub for producing an enormous amount of software and computer programs, but unfortunately, there is no significant Indian contribution in the development of the bioinformatics algorithm. In South Asian countries, the algorithm production is very rare and there is not even a single tool or application which was produced by any South Asian expert [30, 31].

## 8. Comprehensive Platform Framework for the Development of South Asian Bioinformatics Education Database

A comprehensive platform framework is suggested to make a database about the status of South Asian bioinformatics education. The procedure for the development of this system is to form a database, which will store information regarding the status and knowledge of South Asian education from a bioinformatics scenario (Figure 1). The database will be named as SABE (South Asian Bioinformatics Education Database). Users would be able to take search regarding the bioinformatics in South Asian countries and the country name, by the experts of this field and by the university name to explore the top-ranked outputs relevant to queries. This single platform would be available to end users for providing useful updated complete information of South Asian bioinformatics education.

## 9. Suggestions for the Improvement of Bioinformatics Education in South Asia

These are some of the suggestions to improve the prospect of bioinformatics in South Asia:

1. The study of bioinformatics should be made compulsory in all degrees of natural science and along theory; measures must be taken to make the students familiar with practical and dry lab work including molecular modeling, BLAST, gene prediction, gene analysis, and complete protein studies. This will create more opportunities for bioinformatics graduates
2. Short courses and diplomas must be designed for imparting bioinformatics knowledge. These courses would help them to work effectively in a skillful and diverse workforce
3. Seminars must be arranged to create a diverse community having skills in mathematics, statistics, computer science, and biological sciences
4. Because most of the research was undertaken in universities, therefore, students and researchers in universities must be encouraged to attend training and conferences related to bioinformatics
5. Diploma courses are very necessary to make the bioinformatics workforce. In the past, universities like Allama Iqbal Open University (ALU), VU of Pakistan, and Bioinformatics Institute of India had started short courses and distance learning diplomas. But sadly, these courses are now abandoned in Pakistan. Pakistan must have to start their diploma programs again
6. Local universities must collaborate with foreign universities and research institutes. It would increase the worth of a local degree
7. To promote the prospect of bioinformatics, a persuasive campaign must be designed on social media to spread the message of bioinformatics throughout South Asia
8. The bioinformatics curriculum that is taught in South Asian universities should be recognized by the legal education bodies like HEC and BTIS in Pakistan and India, respectively

## 10. Conclusion

Bioinformatics is an interdisciplinary emerging field, and it leads a lot of expertise as it deals with many branches of science. The bioinformatics education started in South Asia with less interest, but the interest is developing among students, governments, industry, and other stakeholders. Bioinformatics can fill the gap of the latest scientific research in South Asia if little extra and dedicated efforts are done by the government. The bioinformatics industry can be a source of income and a source of developing bioinformatics in South Asia. Despite many challenges and problems, bioinformatics is progressing in South Asia with great speed, but this pace of improvement can be accelerated with little more focused struggle by all stakeholders. At the end, based upon the literature review, a framework of the development of a centralized database (SABE) is suggested to collect and store the information on the current status of South Asian bioinformatics education.

## Figures and Tables

**Figure 1:** The schematic representation of SABE framework.

## Supplementary Materials

Supplementary Materials Table 1: some of the major universities in India offering different bioinformatics courses. Table 2: some of the Pakistani universities offering different courses and degrees in bioinformatics. Table 3: universities in Sri Lanka offering bioinformatics degree and courses. Table 4: universities offering bioinformatics courses in Nepal and Bangladesh. Table 5: major conferences and workshops of bioinformatics held in South Asian countries.
